# Ability of visible imaging and machine learning in detection of chickpea flour adulterant in original cinnamon and pepper powders

This article has been retracted.

**DOI:** 10.1016/j.heliyon.2024.e35944

**Published:** 2024-08-08

**Authors:** Mohammad Hossein Nargesi, Kamran Kheiralipour

**Affiliations:** Mechanical Engineering of Biosystems Department, Ilam University, Ilam, Iran

**Keywords:** Adulteration, Image processing, Artificial neural networks, Support vector machine

## Abstract

Adulteration detection in plant-based medicinal powders is necessary to provide high quality products due to the economic and health importance of them. According to advantages of imaging technology as non-destructive tool with low cost and time, the present research aims to evaluate the ability of the visible imaging combined with machine learning for distinguish original products and the adulterated samples with different levels of chickpea flour. The original products were black pepper, red pepper, and cinnamon, the adulterant was chick pea, and the adulteration levels were 0, 5, 15, 30, and 50 %. The results showed that the accuracies of the classifier based on the artificial neural networks method for classification of black pepper, red pepper, and cinnamon were 97.8, 98.9, and 95.6 %, respectively. The results for support vector machine with one-to-one strategy were 93.33, 97.78 and 92.22 %, respectively. Visible imaging combined with machine learning are reliable technologies to detect adulteration in plant-based medicinal powders so that can be applied to develop industrial systems and improving performance and reducing operation costs.

## Highlights

• Chick pea adulterant in black and red pepper and cinnamon was detected.
• Different adulteration levels were evaluated from 0 to 50 %.
• Visible imaging and machine learning methods was used to classify adulteration levels.
• The results of artificial neural network were better than support vector machine.

## 1 Introduction

As quality is one of the main components of sustainable production [1], adulteration controlling has attracted the attention of people and organizations for guaranteeing the quality of different products. Medicinal plants as important products that have been used throughout history required new technologies to detect adulterations. Different plant-based powdered are consumed in traditional medicine, to treat several human diseases. Moreover, according to World Health Organization reports, 70–80 % of the world's population depends mainly on plant-based medicinal materials in medicine and pharmaceuticals health care [[2], [3], [4], [5], [6], [7], [8]].

The main compositions of cinnamon and pepper are moisture, fiber, oil, carbohydrates, protein, vitamins, minerals, alcohol and ash [9]. The products are of plant-based powders that consumed for traditional pharmaceuticals goals. For example, cinnamon prevents the oxidation of organic substances in the body and reduces free radicals due to its strong antioxidant properties. In addition to having anti-inflammatory effects, it is anti-cancer and also has a very strong antimicrobial effect against bacteria, fungi, viruses, and larvae [[10], [11], [12], [13], [14]]. Cinnamon has been used as one of the culinary ingredients in the food industry [15]. In addition, bioactive molecules in cinnamon have been used in the treatment of many diseases and as an insect repellent [[15], [16], [17], [18], [19]]. Pepper is also used as a traditional medicine. Numerous epidemiological studies and interventional trials have shown that pepper can reduce many diseases such as coronary heart disease and cancer. Studies have also confirmed the anti-inflammatory properties of pepper and investigated it against nerve pain and musculoskeletal pain disorders. The health benefits of peppers are the result of various antioxidants and phytochemicals found in peppers [20].

These materials are also consumed as food seasonings not only to enhance the organoleptic properties of food, but also to increase quality and shelf life via reducing or eliminating food pathogens [21,22]. The products are important considering their economic aspect of the products in different countries. However, different materials are mixed with these products as a food adulterant, such as chickpea flour, due to its fast coloring and complete homogenization of the mixture.

Different techniques have been used to detect fraud in different products [23,24] including gas chromatography ion kinetic spectroscopy [25], mass spectrometry [26], NIR [20,27], and NIR and FT-IR fingerprinting [28]. According to high accuracy and speed without need to experts and laboratory materials and operations, visible imaging has been used in different research and application domains [[29], [30], [31], [32], [33], [34]] and also assessment of powdery materials [[35], [36], [37], [38]]. Imaging, preprocessing, feature extraction, and data analysis are the main steps in this technique [30,[39], [40], [41]]. Data analysis is done to predict/classify the obtained features [[42], [43], [44], [45]]. Machine learning methods involving artificial neural network (ANN) [[46], [47], [48], [49], [50]] and support vector machine [[51], [52], [53]].

Rashvand et al. [54] evaluated an olive oil adulteration detection system based on image processing and reported that the classifier predicted the samples with the correlation coefficient of 0.944–0.946 and mean square error of 0.0003–0.006. Different adulterant materials have been detected in previous researches such as cinnamon waste in cinnamon powder [55], stone powder in tapioca starch [56], peanut shell in pepper and cumin [57], talc, rice flour, corn starch, peanut butter powder, and white corn powder in garlic powder [58], and nut shells in cumin powder [59,60]. In the present research, chickpea flour has been considered as an adulterant in powdered plant based medicinal powders. Previously, chickpea flour adulterant has been detected in different products [36] and the local markets proved that it is used as adulterant in cinnamon and pepper.

Considering the advantages of imaging technology and the importance of detecting adulteration in medicinal plants, the purpose of the present research was to evaluate the ability of image processing combined with machine learning methods to detect chickpea flour as adulterant material in three plant-based medicinal powders as red and black pepper and cinnamon. Two methods were used to analysis the data and their results were compared to reach higher accuracy.

## 2 Materials and methods

### 2.1 Samples preparation

The original pure black and red pepper seeds and cinnamon rhizome were purchased in local markets, Ilam, Iran, as base material of medicinal plants. The purchased materials were grinded using a regular blade grinder to obtain plant-based medicinal powders (Fig. 1). Chickpea flour was used as adulterant material [55]. It was purchased from the markets. A 300-μm mesh sieve was used to filter the powders. Chemical methods were not used to checked the authenticity of the samples.

**Fig. 1:** The origin samples including black pepper (a), red pepper (b), and cinnamon (c), and powdered samples including black pepper (d), red pepper (e), and cinnamon (f), and powdered adulterant (chickpea) (g).

To prepare adulterated samples, chickpea flour was used to be mixed with the plant-based medicinal powders. Five adulteration levels of 0, 5, 15, 30, and 50 % (by weight) were obtained. The samples were stored separately in closed plastic bags in a cool, dark, and dry environment. One sample of each adulteration level has been presented in Fig. 2. Three samples were provided for each adulteration level and six images were provided for each sample.

**Fig. 2:** Different adulteration levels of the plant-based medicinal powders.

### 2.2 Imaging and image processing

The samples were photographed using the Xiaomi Note 10 Pro camera (Fig. 3). For imaging the samples, 10 g of each sample was placed in the imaging system. For each adulteration level, 18 images were taken from each sample, so that total of 270 visible (RGB) images were acquired from the samples. The images were used as input to the image processing algorithm.

**Fig. 3:** Different conducted steps in the present research from imaging to classification.

An image processing algorithm was developed in MATLAB R2016b software to process the acquired images of the adulterated medicinal powder samples. The first step of visual image processing is to provide a useful image in order to extract features. The improvement of the images was done through the segmentation of the useful areas of the images [61]. In the present research, the center of the image was cropped to be used to extract color and textural features of the image [47].

Feature extraction was done in order to calculate different parameters from the cropped parts of the image. The extracted features included color and textural features from the images of the samples. Minimum, median, mean, coefficient of variation, mode, standard deviation, kurtosis, and skuness were calculated as color features. The extracted textural features include energy, contrast, entropy, correlation, and homogeneity [62].

As great number of features extracted from the images (266 features) need more time for classification and may lead to decrease detection accuracy, so a few of them were selected as efficient features. The more the difference between the efficient features of the adulteration level, the more the classification accuracy. So, only the efficient features were used for classification. An algorithm was designed and codded in MATLAB software to find the efficient features based on the sequential feature selection method. In the algorithm, the inputs were the extracted features and the output were the classes. The used method selects the features based on the of the deviance of the fit (a generalization of the residual sum of squares) criterion.

### 2.3 Classification

Artificial neural networks and support vector machine methods have been used to classify the efficient features. ANN is one of the most effective machine learning algorithms that is widely used as an artificial intelligence approach for data analysis [63,64]. The back-propagation feed forward ANN type was used with Levenberg-Marquardt training model due to its high accuracy and speed, as well as to prevent network overtraining [41,46]. The activation functions in both hidden and output layers was tansig. for ANN classification, 60 % of the data was used in training, 20 % for validation, and 20 % for test step. In SVM classification, 80 % of the data was used in training and 20 % in test step.

## 3 Results and discussion

### 3.1 Efficient features

The total number of features extracted from the visible images was 266, due to the abundance of the feature and the possibility of causing errors in the classification results, the effective features were selected and then used as the input of the classification model (Table 1). In this research, 14, 14, and 16 features were selected as efficient features of black pepper, red pepper, and cinnamon powders, respectively.

**Table 1:** The mean of the efficient features of different classes of pepper and cinnamon.

Based material	Feature	Channel	Adulteration level				
			0 %	5 %	15 %	30 %	50 %
Black pepper	Mean	Gray	0.47	0.49	0.51	0.54	0.59
	Median	Gray	0.50	0.53	0.56	0.60	0.65
	Median	Red	0.58	0.60	0.63	0.67	0.72
	Mean	Blue	0.33	0.35	0.36	0.38	0.41
	Median	a*	4.06	3.13	2.39	1.57	0.80
	Mean	b*	22.36	21.86	22.76	22.48	22.89
	Mean	i1	0.45	0.46	0.48	0.51	0.55
	Coefficient of variation	i2	0.21	0.20	0.21	0.20	0.16
	Mean	i3	0.01	0.01	0.02	0.02	0.03
	Standard deviation	Cg	0.01	0.01	0.01	0.01	0.01
	Mode	Cb	−0.16	−0.15	−0.17	−0.18	−0.19
	Energy	Hue	0.84	0.72	0.58	0.46	0.41
	Entropy	Saturation	6.90	7.03	7.05	6.98	6.91
	Median	Value	0.58	0.60	0.63	0.67	0.72

Red pepper	Mean	Gray	0.41	0.42	0.45	0.52	0.59
	Entropy	Gray	7.48	7.51	7.57	7.56	7.49
	Homogeneity	Gray	0.71	0.79	0.70	0.70	0.70
	Skewness	Blue	0.48	0.42	0.32	0.17	−0.15
	Mean	L*	66.82	67.79	69.79	74.60	79.50
	Median	b*	70.01	66.23	54.70	40.39	26.92
	Energy	Ng	0.38	0.42	0.51	0.52	0.68
	Entropy	i1	7.32	7.36	7.45	7.47	7.45
	Median	i1	0.37	0.39	0.42	0.51	0.59
	Contrast	I3	1.01	1.05	1.22	1.35	1.30
	Energy	b*	0.39	0.32	0.20	0.12	0.08
	Standard deviation	Cb	0.14	0.14	0.12	0.08	0.04
	Coefficient of variation	Hue	0.42	0.40	0.34	0.24	0.15
	Entropy	Hue	7.65	7.66	7.67	7.54	7.40

Cinnamon	Mean	Gray	0.43	0.43	0.43	0.46	0.50
	Median	Gray	0.46	0.45	0.46	0.49	0.54
	Energy	Gray	0.06	0.05	0.06	0.05	0.05
	Energy	Red	7.51	7.60	7.61	7.63	7.61
	Median	Red	0.65	0.64	0.65	0.66	0.69
	Mean	Blue	0.15	0.15	0.16	0.19	0.24
	Median	a*	4.05	12.65	12.39	10.69	8.13
	Coefficient of variation	b*	0.62	0.37	0.37	0.40	0.46
	Mean	i1	0.49	0.38	0.39	0.41	0.46
	Entropy	i1	7.58	7.38	7.39	7.47	7.54
	Energy	i11	0.05	0.06	0.06	0.06	0.05
	Mode	Cr	0.07	0.18	0.18	0.16	0.14
	Mean	Saturation	0.48	0.80	0.80	0.76	0.68
	Median	Saturation	0.38	0.78	0.78	0.72	0.62
	Skewness	Value	−0.10	−0.04	0.02	−0.20	−0.04
	Correlation	Value	0.74	0.71	0.73	0.74	0.76

In Table 1, the number of efficient features were selected for the studied products. The result shows that the values of those features were different for different levels of adulteration. According to the data in Tables 1 and it can be found that with the increase in the percentage of adulteration, the difference between the values of the efficient features increases. The average values of the efficient features for the adulteration level of 50 % were the highest values for almost all the features. Also, the highest average values for median of a*, coefficient of variation of i2, and energy of hue channels can be seen in pure black pepper. Table 1 shows that the average values of 14 efficient features of red pepper are different for different classes. The average features of skewness of blue, median and energy of b*, standard deviation of Cb, and variation coefficient of channels were the highest for pure red pepper. The values of other efficient features were highest for other adulteration levels. From the data in Tables 1 and it can be found that the average values of 16 effective features for cinnamon are different in different adulteration levels. The median of all efficient features for the 50 % adulteration level was the highest except for the averages of energy of gray, variation coefficient of b*, and mean and entropy of i1 channels which had the highest values for pure cinnamon.

### 3.2 Classification

#### 3.2.1 Support vector machine

The results of the classifier based on SVM method with one-against-one strategy for adulteration detection in the studied products has been presented in Fig. 4. The classifier correctly identified all samples in the third, fourth, and fifth classes as black pepper with 15, 30, and 50 % adulteration of chickpea flour, respectively. Three and two samples corresponding to pure samples and 5 % adulteration corresponding to the first and second class, respectively, were classified incorrectly. According to the confusion matrix obtained for the support vector machine classifier, 85 out of 90 samples were correctly recognized and 5 samples were wrongly detected. The correct classification rate of this classifier model was equal to 93.33 %. All the studied samples were correctly identified by the classifier, except for 2 samples from the first class, which are related to pure red pepper. According to the results of the support vector machine classification, the correct classification rate was 97.78 %. The classification has been done correctly for all classes, except for class number 2, which is related to cinnamon with 5 % chickpea flour adulteration. According to the confusion matrix, 87 out of 90 samples were correctly identified and only three samples were misclassified. So, the correct classification rate of the classifier was 92.22 %.

**Fig. 4:** The classification results of the SVM model to classify adulteration levels of chickpea flour in the studied products.

#### 3.2.2 Artificial neural networks

In order to classify different levels of adulteration of chickpea flour in black pepper, different models were investigated and evaluated based on ANN method. For this purpose, the number of neurons in the hidden layer has been changed to evaluate different classification structures. The number of neurons in input and output layer were equal to the number of efficient features and the number of adulteration levels, respectively. Based on the correct classification rate, the best classification model of black pepper with chickpea flour adulteration was selected.

To detect different levels of adulteration of chickpea flour in black pepper, the optimal network had 14-10-5 structure. In this structure, 10 neurons were obtained for the hidden layer (Fig. 5a). Fig. 6 shows the classification results of the optimal ANN model in classification of different levels of fraud in black pepper. According to the matrix, all samples were correctly identified except for the second and fourth classes, which correspond to fraud levels 5 and 30 % adulteration, respectively. Based on this, it can be reported that 88 out of 90 samples have been correctly classified so that classification accuracy was 97.8 %. The validation performance of the optimal artificial neural network classifier has been shown in Fig. 7a. As seen, the lowest error in the validation step was obtained in epoch number 8 with an error of 0.035852. Fig. 8a shows the correlation coefficients (r) of the optimal artificial neural network classifier for training, validation, test, and all data. The coefficient with power of two (r^2^) is the prediction accuracy of the classes. It can be seen that the correlation coefficient of the optimal network for training, validation, test and all data was equal to 97.61, 88.15, 97.21, and 95.65 %, respectively.

**Fig. 5:** The optimal structure of artificial neural network model for classify different adulteration levels of black pepper (c), red pepper (b), and cinnamon (c).

**Fig. 6:** The classification results of the ANN model to classify adulteration levels of chickpea flour in black pepper (c), red pepper (b), and cinnamon (c).

**Fig. 7:** The validation performance of the optimum classifier for adulteration detection of chickpea flour in black pepper (c), red pepper (b), and cinnamon (c).

**Fig. 8:** The regression results of the optimal ANN for classification of adulteration levels in black pepper (c), red pepper (b), and cinnamon (c).

The optimal artificial neural network structure was 14–10-5 for detecting adulteration of chickpea flour in red pepper. The number of neurons in the input layer was 14, the number of neurons in the hidden layer was 10, and the number of neurons in the output layer was 5 (Fig. 5b). The classification results of the optimal model based on artificial neural network method for the detection of chickpea flour in red pepper was shown in (Fig. 6). The classification accuracy of the optimal structure was 98.9 %. Fig. 7b shows the performance of the network in the validation step for the number of different epochs. The best network validation performance occurred in epoch number 13 with a mean square error of 0.10291. The correlation coefficients for the optimal model for training, validation, testing, and all data were 99.93, 96.78, 94.27, and 98.19 %, respectively (Fig. 8b).

The optimal artificial neural network classifier for classifying different levels of cinnamon adulteration had a 16-15-5 structure. the ANN model had 16 neurons in the input layer, 15 neurons in the hidden layer, and 5 neurons in the output layer (Fig. 5c). The classification results of the classifier for different levels of chickpea flour adulterant in cinnamon powder has been shown in Fig. 6. The result showed that the correct classification rate of adulteration detection was 95.60 %. The result means that the classifier correctly recognized all the samples in the first, fourth, and fifth classes, but it wrongly recognized 4 samples that belong to the second and third classes. Now the classifier has been able to recognize 86 out of 90 samples. Validation performance of the optimal network for classification different adulteration levels of red pepper had been shown in Fig. 7c. In epoch number 9, the lowest error has been observed as 0.032114. Fig. 8c shows the correlation coefficients of the optimal neural network model for training, validation, testing and the all data. The correlation coefficients of the optimal classifier for the data sets were 96.37, 89.47, 85.56, and 92.87 %, respectively.

The classification accuracies of the classifier based on support vector machine method with one-against-one strategy to detect different levels of chickpea adulterant in black pepper, red pepper, and cinnamon powders were 93.33, 97.78, 92.22 %, respectively. Whereas, the accuracies of the classifier model based on artificial neural networks method for classifying different adulteration levels in the powders were 97.8, 98.9, and 95.6 %, respectively. The classification accuracies of the two used methods for red pepper were higher compared to other products this fact is due to higher difference between the color of red pepper and chickpea powders. The lowest accuracies of the two methods were obtained for cinnamon which is due to lower diffidence between the color of cinnamon and chickpea powders.

The accuracy of artificial neural network and support vector machine in classifying adulteration levels in the present research was higher than previous studies. Mohammadzadeh Moghadam [51] classified saffron based on color characteristics. The results of their research showed that the average accuracy using SVM classifier was 82.23 %. These shows higher ability of the proposed framework in the present research to detect different adulteration levels in the studied products.

As original grain samples were purchased from the local markets, the authority of the samples were not checked. However, for industrial applications of the framework there is needed to conduct chemical tests to prove the authority of the samples.

## 4 Conclusions

In this research, adulteration detection of chickpea flour in three types of *original* plant-based medicinal powders including black pepper, red pepper, and cinnamon were investigated using visible imaging. Efficient color and textural features were selected for 0, 5, 15, 30, and 50 % adulteration levels. The classification accuracy of machine learning methods including artificial neural network and support vector machine methods were evaluated. The accuracies of the ANN model (97.8, 98.9 and 95.6 %, respectively) were higher than those of SVM classifier (93.33, 97.78 and 92.22 % respectively). There can be concluded that visual image processing combined with artificial neural network can be used to for classification of adulteration levels and development of automatic detection systems. According to high speed and accuracy without needs to experts and laboratory materials and operations, visible imaging is a non-destructive powerful technique in quality assessment of medicinal plants and powders.

Moreover, other classification techniques can be applied in future research to increase classification accuracy of the detection of adulteration in the studied food materials. Other imaging techniques such as hyperspectral imaging can be used to improve the results in future.

As, the goal of the present research was to evaluate the ability of the proposed framework including imaging and machine learning for distinguish original products and the adulterated samples with different levels of chickpea flour, the authenticity of the products was proved by a local market. So, the *authenticity* of the samples was not checked using chemical methods. However, for industrial applications of the proposed framework, it is recommended to measure the component of the main products to check their authenticity. Also, it is recommended to study large variety of samples with different geographical, harvest seasons, and spiked with other adulterants to provide a reputable source to develop a robust machine vision system for detect different adulterants and estimate different adulteration levels in the studied products.

## CRediT authorship contribution statement

**Mohammad Hossein Nargesi:** Writing – original draft, Formal analysis, Data curation. **Kamran Kheiralipour:** Writing – review & editing, Software, Resources, Formal analysis.

## Declaration of Competing interest

The authors states there is no declaration of interests in the present manuscript.
